# Estimating the Impacts of Hospitals' Organisational and Geographical Characteristics on the Adoption of Health Information Technology in Mongolian Hospitals

**DOI:** 10.1155/2021/8836625

**Published:** 2021-05-10

**Authors:** Sarnai Tsagaankhuu, Enkhdulguun Amgalan, Turtushikh Damba, Xinping Zhang

**Affiliations:** ^1^School of Medicine and Health Management, Tongji Medical College, Huazhong University of Science and Technology, Wuhan, China; ^2^Division of University Hospital Development, Mongolian National University of Medical Sciences, Ulaanbaatar, Mongolia; ^3^School of Public Health, Mongolian National University of Medical Sciences, Ulaanbaatar, Mongolia; ^4^Department of Pharmaceutical Chemistry and Pharmacognosy, School of Pharmacy, Mongolian National University of Medical Sciences, Ulaanbaatar, Mongolia

## Abstract

**Background:**

The adoption of health information technology (HIT) is an important measure for improving healthcare quality and safety, which is affected by many hospital factors, but it has not yet been estimated in the Mongolian hospital sectors. This study examines how hospitals' organisational and geographical characteristics influence the adoption of HIT in Mongolian tertiary and secondary care hospitals.

**Methods:**

А cross-sectional study involving the executive directors and medical equipment engineers was conducted in 39 hospitals. Data acquired from questionnaires are (1) hospitals' organisational and geographical characteristics, including bed-size capacity, ownership type, status, and location of the hospitals, and (2) the adoption rate of HIT, and its categories are based on the Health Information and Management Systems Society's classification (2002). The dependent variable was measured as numbers and the rate of HIT programs adopted clinical, administrative, and strategic information technologies (IT). A regression analysis was used to estimate the factors of impact on the adoption of clinical, administrative, and strategic IT.

**Results:**

We found a concerning relationship between the characteristics and adoption of HITs. On average, the number of HIT programs adopted was 18, covering nine clinical IT programs, six administrative IT programs, and three strategic IT programs. The adoption rate of overall HIT was 33.29% in the hospitals. In regression analysis, the organisational and geographical characteristics' impact and HIT adoption of hospitals was positively associated with large bed-size (clinical IT: *β* = 0.256, *P* < 0.001; administrative IT: *β* = 0.3654, *P* < 0.001; strategic IT: *β* = 0.0006, *P* < 0.001), for-profit (strategic IT: *β* = 0.1995, *P* < 0.01), teaching (clinical IT: *β* = 0.2560, *P* < 0.05; administrative IT: *β* = 0.1985, *P* < 0.05; strategic IT: *β* = 0.2236, *P* < 0.01), and urban location (clinical IT: *β* = 0.2840, *P* < 0.001, administrative IT: *β* = 0.2256, *P* < 0.01; strategic IT: *β* = 0.2256, *P* < 0.001).

**Conclusion:**

Our study found that the HIT adoption rate in Mongolia is poor, and its adoption is mainly positively associated with bed-size capacity, status, and location of the hospitals. Also, we found that the ownership type is partially affected HIT adoption.

## 1. Introduction

Health information technology (HIT) is an important tool for improving healthcare quality and patient safety [1]. In HIT sector, many studies have been conducted in developed countries, while little is known in developing countries. Mongolian healthcare system was inherited from the former Soviet centralized Semashko system and underwent modifications over time [2].

The system consists of two tiers: primary and referral level care. Primary level care is delivered by family health centre, soum (a country subdivision) health centre, and inter-soum hospitals. People who seek medical attention first go to primary level care, and in case the sickness could not be diagnosed or treated, they would go to referral level care which provides specialized care. Whereas, secondary and tertiary care facilities provide the referral level care in Mongolia. If secondary care hospital could not provide a healthcare, patients have to seek medical services from tertiary care hospital. Tertiary care hospitals provide high level of multispecialty care in the capital of Mongolia, Ulaanbaatar [3, 4]. Hospital classification of Mongolia is shown in Figure 1.

In Mongolia, the health insurance law was approved in 2015, and it was principally focused on the gatekeeper role of primary care similar to the UK system. However, the law reformed again for the Taiwan model which was based on performance and patient choice of facilities in 2021 [5].

Mongolian public hospitals are financed from the state budget, the health insurance fund, and client fees. Public hospitals mostly serve poor lower middle-income people, who make up about 60% of the total population, whereas higher income citizens tend to seek care from private hospitals or abroad. Thus, improving public hospital management is beneficial to the poorer and lower middle-income groups. The public healthcare sector accounts for 78% of total hospital beds and 80% of total hospital admissions and absorbs nearly 70% of the national health budged [6]. According to 2018 statistics, 28.4 percent of Mongolia's population lives in poverty [7]. HIT is a fundamental measure for the improvement of healthcare delivery [8]. Currently, there are no studies or evidences published about the Mongolian hospitals which have not fully adopted electronic medical records. According to the accountable specialists, only 3 tertiary and 2 secondary care hospitals have applied electronic medical record, but only in outpatient wards, whereas four private hospitals have fully applied electronic medical record and are leading the application of electronic medical records in the country. In addition, a significant number of healthcare providers still store patient records on paper documentation [9].

HITs are reported to enhance patient safety by reducing complications and mortality rates, as well as by minimizing medical errors covering clinical, administrative, and strategic information technologies [10]. However, HIT is able to prevent medication errors in many ways, and it may also potentially introduce new paths to errors. Wang et al. studied 152 reports of medication errors caused by HIT. The study found that 64.93% of them were due to errors in health information technology [11].

The aim of our research was to determine the relationships between a hospital's (organisational and geographical) characteristics and the adoption rate of HIT in Mongolian tertiary and secondary care hospitals.

## 2. Research Framework and Hypothesis

We applied *Avedas Donabedian*'*s* the “Structure-Process-Outcome” conceptual model on to the dominant theoretical model in health services research. This conceptual model analyses the quality of healthcare from three dimensions: structure, process, and outcome [12]. According to this model, the quality of the healthcare system can be defined along three dimensions. “Structure” is the system's material, organisational, and human resources. “Processes” are the activities performed by the system and its people, such as healthcare delivery methods. “Outcomes” are the measurable end results, such as mortality, patient health status, and medical error rates [13]. Due to the limited information, we only conduct the link between “structure” and “processes.”

Based on the results of previous studies [14, 15], we hypothesized relationship between the organisational and geographical characteristics, and the adoption rate of HIT is illustrated below:

  H1 Larger hospitals will adopt HIT more extensively than smaller hospitals.
  H2 Teaching hospitals will adopt HIT more extensively than nonteaching hospitals
  H3 For-profit hospitals will adopt HIT more extensively than not-for-profit hospitals
  H4 Urban hospitals will adopt HIT more extensively than rural hospitals

## 3. Materials and Methods

А cross-sectional study was conducted in 39 hospitals by asking the executive directors and medical equipment engineers. The setting included 34 secondary care hospitals, which are district and provincial hospitals administered by an agency of district or provincial governments, and five tertiary care hospitals are owned by an agency of state that located in capital of Mongolia. Data acquired from questionnaires are (1) hospitals' organisational and geographical characteristics, including bed-size capacity, ownership type, status and location of the hospitals and (2) the adoption rate of HIT, and its categories are based on the Health Information and Management Systems Society's classification (2002). The dependent variable was measured as numbers and the rate of HIT programs that adopted clinical, administrative, and strategic information technologies (IT). A regression analysis was used to estimate the factors of impact on the adoption of clinical, administrative, and strategic IT.

### 3.1. The Definition and Measurement of the Hospital Characteristics

Characteristics consist of organisational (hospital bed-size capacity, status, and ownership type) and geographical (location).

#### 3.1.1. Hospital Bed-Size Capacity

According to the World Health Organization's classification, hospitals can be divided as three groups based on the hospital bed-size capacity that having up to 100 beds are considered as small, more than 100 to less than 300 beds are medium, and more than 300 beds are large hospitals, respectively [16].

#### 3.1.2. Hospital Status

All hospitals were placed into 1 of 3 categories based on their response to the American Hospital Association survey: major teaching hospitals, minor teaching hospitals, and nonteaching hospitals (all other institutions). As there are no major teaching hospitals in Mongolia, the concept of teaching hospitals, includes hospitals affiliated to medical university [17].

#### 3.1.3. Ownership Type

Two types of ownership are analyzed in this study: for-profit and not-for-profit [18] hospitals including affiliated with state-owned enterprises. Also, some private hospitals' ownership is not-for-profit in Mongolia.

#### 3.1.4. Location

Geographical characteristic refers to each *hospitals*' *location* (urban/rural) [17].

### 3.2. The Definition and Measurement of the Adoption of HIT and Its Categories

The HIT categories were formulated from a list compiled by the Health Information and Management Systems Society (2002) leadership survey and was further refined based on an extensive literature review and consultations with HIT experts [19]. It includes three categories:

 
*Clinical IT* consists of systems designed to improve patient care, such as computerized physician order entry systems, electronic medical records, and pharmacy information systems
 
*Administrative IT* includes applications intended to streamline and improve internal data processing activities, such as patient registration systems, billing systems, and payroll processing systems
 
*Strategic IT* includes applications intended to improve critical decision-making activities, such as managed care software, nurse staffing systems, and executive information systems

Our dependent variable was measured as a raw count (frequency) and rate (%) of HIT applications checked by respondents and individual counts of applications as well as checked within each application cluster (clinical, administrative, and strategic IT).

The clinical IT programs scale ranged from 0 (no clinical IT) to 25 (all 25 clinical IT items implemented). Likewise, the administrative IT programs scale ranged from 0 to 18, and the strategic HIT scale programs ranged from 0 to 9. The overall IT adoption index, created by summing up the three component scales programs, ranged from 0 to 52 for each hospital.

### 3.3. Statistical Analysis

Statistical analysis was performed using SAS 9.1 software. The negative binomial regression was used to identify the organisational and geographical characteristics that impact the adoption of clinical, administrative, and strategic IT in Mongolian hospitals.

## 4. Results

### 4.1. Organisational and Geographical Characteristics

Hospitals were divided, based on the number of hospital bed-size capacity, into the three groups: seventeen of the hospitals' bed-size capacity were small (43.5%) and 17 were medium (43.5%), whereas only five hospitals (12.8%) were categorized as large.

Nearly two-thirds (64%) of the hospitals were located in rural areas, while 36% were located in urban areas. A majority of the hospitals were nonteaching (76.9%) and not-for-profit (87.2%). See Table 1, for details.

On average, the number of HIT programs that are adopted by hospitals reached 18, of which nine were clinical IT programs, six were administrative IT programs, and three were strategic IT programs. The overall adoption rate ranged between 29.02 and 38.05% with a mean of 33.29%. It indicates that less than half of all Mongolian hospitals adopted the three clusters of technologies at the time of the survey, as shown in Table 1. The average levels of adoption for each technological category were consistently higher at large bed-size hospitals in comparison to those medium and small bed-size hospitals. On average, large bed-size hospitals adopted 13.47 clinical programs, 7.17 administrative programs, and 5.35 strategic programs, whereas medium bed-size hospitals adopted 9.25 clinical programs, 5.36 administrative programs, and 4.17 strategic programs. In small bed-size hospitals, 8.89 clinical programs, 3.25 administrative programs, and 1.25 strategic programs were adopted. Large bed-size hospitals were more than twice the adoption rates (50.75%) in comparison to small bed-size hospitals (23.18%).

For-profit hospitals' adoption rates were 11.6 clinical programs, 6.7 administrative programs, and 4.14 strategic programs, compared to the not-for-profit adoption rates of 8.45 clinical programs, 5.85 administrative programs, and 2.10 strategic programs. Therefore, for-profit hospitals were higher adoption rates of HIT (43.2%) than not-for-profit hospitals (29.87%).

Teaching hospital's adoption rates (10.54 for clinical, 5.28 for administrative, and 4.78 for strategic technologies) were higher than nonteaching hospitals (7.18 for clinical, 4.46 for administrative, and 1.81 for strategic technologies. This result showed that teaching hospitals were higher IT adoption rates (41.53%) than non-teaching hospitals (24.53%).

Finally, urban hospitals had a higher technology adoption rate (30.42%) than rural hospitals (13.42%).

Regression analysis for organisational and geographical characteristics showed impact on rate of HIT adoption. In the result, organisational and geographical characteristics were impacted on the adoption of clinical technologies.

We examined the relationship between each element of the healthcare IT cluster and the hospitals' organisational and geographical characteristics. The adoption of clinical technologies in Mongolian secondary and tertiary care hospitals were positively associated with bed-size (*P* < 0.001), location (*P* < 0.001), and teaching status (*P* < 0.05) of the hospitals, see Table 2.

As can be seen from Table 2, administrative IT was positively affected by bed-size (*P* < 0.001), urban location (*P* < 0.01), and teaching status (*P* < 0.01) of the hospitals. However, ownership type did not appear to affect the adoption of administrative technologies. And, the adoption of strategic IT was positively associated with bed-size (*P* < 0.001), urban location (*P* < 0.001), and ownership type (*P* < 0.01). Hospital location did not significantly impact the adoption of strategic IT.

The hypothesis H3 was partly rejected, whereas the hypotheses H1, H2, and H4 were accepted (*P* < 0.05).

## 5. Discussion

Our findings support that the HIT adoption rate is poor in Mongolian hospitals and HIT adoption positively associated with hospital bed-size capacity, status, and location of the hospitals. In addition, for-profit hospitals were positively associated to the strategic IT adoption.

In Mongolia, the adoption rate of HIT ranged from 29.02% to 38.05%, with a mean of 33.29%. Compared to developed countries, the average adoption rate of HIT was much lower. For example, in Florida's hospitals, mean rate of HIT adoption was found to be higher (clinical IT 45%, administrative IT 74% strategic IT 50%, and mean HIT adoption rate 57%) than Mongolian hospitals' adoption rate. A study conducted in the United States of America reported a 50% failure rate for clinical technology implemented in healthcare organisations [20].

From the organisational characteristic perspective, we found that the hospital bed-size capacity was the most important predictor of the adoption of all three HIT. Large bed-size hospitals consistently adopted the largest number of clinical, administrative, and strategic IT programs compared to small and medium bed-size hospitals. These results are similar to the previous findings that Neset et al. also found positive associations between hospital bed-size capacity and adoption of clinical and strategical IT, but not with administrative IT [20]. This implies that large bed-size hospital is positively associated with adoption of HIT, but may vary between the type of IT.

We also found that the ownership and status of hospital were influencing factors of the adoption of HIT. However, only the ownership of hospital had no effect on clinical IT. Lee et al. reported that the rate of clinical IT adoption differs in degree by hospital characteristics. Large bed-size, teaching, and for-profit hospitals were closely related to clinical IT adoption, while teaching, not-for-profit, and large bed-size hospital had higher clinical IT adoption rate [21]. This implies that while large bed-size is a relative positive factor in IT adoption, for-profit status is not. Mongolian hospitals are also classified as public or private according to their ownership. For-profit hospitals had significant differences in medical cost. Therefore, they are observed to develop more rapidly in for-profit hospitals. The insignificant result can also be found in other studies. For example, researchers also show that for-profit hospitals significantly affected the adoption of clinical and strategic IT, but not administrative IT. Neset et al. showed that hospital ownership type and status are a significant effect on administrative and strategical, but not on the clinical IT [20]. DesRoches et al. and Upadhyay et al. report that teaching hospitals have the higher level of strategical IT compared to nonteaching hospitals [22, 23].

From the geographical characteristic perspective, our analysis suggested that urban location was the most important indicator of the adoption of all categories of HIT. This suggestion confirms some of the findings of other studies [24], but some highly developed countries results were different from ours. For example, Neset et al. examined whether geographical characteristics influenced adoption of HIT in 98 hospitals in Florida and reported that geographical location was not a significant predictor of HIT adoption [20]. Hospitals in urban areas have better opportunities to collaborate with various industries, government agencies, and institutions of higher education and research, which give possibilities to secure external financial resources and acquire information about these relatively new HIT technologies. Mongolia is considered to be one of the sparsest populated countries in the world in terms of population density, and it was estimated 2 people per square kilometers as for 2019. The population density of the capital city Ulaanbaatar has reached 312.6 per square kilometers in 2019, an increase of 16 (5.2%) compared to previous 5 years [4]. The development of the healthcare sector is not adequate due to its sparse population in rural areas. Mongolia's long-term development policy states to support the introduction of advanced health technologies [7].

Additionally, Ingebrigtsen et al. conducted a systematic review to examine the evidence of associations between clinical leadership and successful information technology (IT) adoption in healthcare organisations. Their results show that clinical leaders who have technical informatics skills and prior experience with IT program management are likely to develop a vision that comprises a long-term commitment to the use of IT. This leads to proactive leadership behavior and partnerships with IT professionals that are associated with successful organisational and clinical outcomes [25]. This study has empirically demonstrated that among Mongolian tertiary and secondary care hospitals, hospital bed capacity, ownership type, and hospital location play a significant role in motivating the adoption of various HIT applications.

## 6. Conclusion

Our study found that the HIT adoption rate is poor compared with developed countries. And, the adoption of all three HIT is mainly positively associated with bed-size capacity, status, and location of the hospitals in Mongolia. Also, we found that the ownership type is partly affected administrative and strategic IT adoption. This study confirmed that organisational and geographical characteristics (structure) impact the adoption of HIT (process), which implies that modifying organsational construction and promoting geographical access (structure) may impact on the adoption of HIT (process). Our suggestion is to enhance hospitals with these structural attributes conducive to more HIT adoption especially for developing countries. The influence of structural attributes on the type of HIT adoption should be generalized with caution.

## 7. Limitations

This study has some limitations that are worth mentioning. The current study focused only on organisational and geographical characteristics' impact on the adoption rate of HIT without considering clinical leadership, due to the unavailability of the data and the limitations of paper length.

In addition, due to limited information, we were not able account the medication error and patient healthcare outcome impact on adoption of HIT. We only performed the analysis of binary categories because of the limited sample size. In the future, we will address these characteristics' impact on the adoption rate of HIT and their impact on medical quality, as well as conducting a national-level study to fully explore the role of individual characteristics on hospitals' HIT adoption rate and medical quality.

## Figures and Tables

**Figure 1:** Mongolia's classification of hospitals.

**Table 1:** Distribution of organisational and geographical adoption rate of HIT in Mongolian secondary and tertiary care hospitals.

Variables	Clinical		Administrative		Strategic		Total
	Number	Rate (%)	Number	Rate (%)	Number	Rate (%)	Rate (%)
Bed-size capacity							
Small (43.5%)	8.89	35.56	3.25	18	1.5	16	23.18
Medium (43.5%)	9.25	37	5.36	29.7	4.17	46.3	37.66
Large (12.8%)	13.47	53	7.17	39.83	5.35	59.44	50.75

Ownership type							
Not-for-profit (87.2%)	8.45	33.8	5.85	32.5	2.1	23.33	29.87
For-profit (12.8%)	11.6	46.4	6.7	37.22	4.14	46	43.2

Status							
Teaching(23.1%)	10.54	42.16	5.28	29.33	4.78	53.11	41.53
Nonteaching (76.9%)	7.18	28.72	4.46	24.77	1.81	20.11	24.53

Location							
Urban (36%)	10.99	43.6	7.02	39	0.78	8.66	30.42
Rural (64%)	4.25	17	1.25	6.94	1.47	16.33	13.42
Frequency of HIT adoption	9		6		3		18
Adoption rate of HIT (%)	38.05		29.02		32.8		33.29

**Table 2:** Multiple regression analysis of the organisational and geographical characteristics on the adoption of HITs.

Variable	Clinical		Administrative		Strategic	
	*β*	95% CI	*β*	95% CI	*β*	95% CI
Bed-size capacity	0.256^*∗∗∗*^	0.2325, 0.2803	0.3654^*∗∗∗*^	0.3452, 0.3856	0.0006^*∗∗∗*^	0.0007, 0.005
Ownership type	0.0456	0.0396, 0.0516	0.0352^*∗∗∗*^	0.009, 0.061	0.1995^*∗∗*^	0.098, 0.301
Status	0.2560^*∗*^	0.1215, 0.4505	0.1985^*∗*^	0.179, 0.218	0.2236^*∗∗*^	0.1512, 0.296
Location	0.2840^*∗∗∗*^	0.1427, 0.4253	0.2256^*∗∗*^	0.1227, 0.3285	0.2256^*∗∗∗*^	0.1489, 1.488

^*∗*^ *P* < 0.05, ^*∗∗*^*P* < 0.01, and ^*∗∗∗*^*P* < 0.001.

## Data Availability

The data used to support the findings of the study are available from the corresponding author upon request.

## Abbreviations

HIT: Health information technology
IT: Information technology.
